# Recognition of Diabetic Retinopathy with Ground Truth Segmentation Using Fundus Images and Neural Network Algorithm

**DOI:** 10.1155/2022/8356081

**Published:** 2022-09-29

**Authors:** Pravin R. Kshirsagar, Hariprasath Manoharan, Pratiksha Meshram, Jarallah Alqahtani, Quadri Noorulhasan Naveed, Saiful Islam, Tewodros Getinet Abebe

**Affiliations:** ^1^Department of Artificial Intelligence, GH Raisoni College of Engineering, Nagpur, Maharashtra, India; ^2^Department of Electronics and Communication Engineering, Panimalar Engineering College, Poonamallee, Chennai, India; ^3^Department of Information Technology, MPSTME Shirpur, Savalade, Maharashtra, India; ^4^College of Computer Science and Information Systems, Najran University, Najran 61441, Saudi Arabia; ^5^College of Computer Science, King Khalid University, Abha 61413, Asir, Saudi Arabia; ^6^Civil Engineering Department, College of Engineering, King Khalid University, Abha 61421, Asir, Saudi Arabia; ^7^Department of Chemical Engineering, College of Biological and Chemical Engineering, Addis Ababa Science and Technology University, Addis Ababa, Ethiopia

## Abstract

Diabetes problems can lead to a condition called diabetic retinopathy (DR), which permanently damages the blood vessels in the retina. If not treated, DR is a significant cause of blindness. The only DR treatments currently accessible are those that block or delay vision loss, which emphasizes the value of routine scanning with high-efficiency computer-based technologies to identify patients early. The major goal of this study is to employ a deep learning neural network to identify diabetic retinopathy in the retina's blood vessels. The NN classifier is put to the test using the input fundus image and DR database. It effectively contrasts retinal images and distinguishes between classes when there is a legitimate edge. For the resolution of the problems in the photographs, it is particularly useful. Here, it will be tested to see if the classification of diabetic retinopathy is normal or abnormal. Modifying the existing study's conclusion strategy, existing diabetic retinopathy techniques have sensitivity, specificity, and accuracy levels that are much lower than what is required for this research.

## 1. Introduction

Diabetes is a determined organ disease that occurs when the pancreas of an individual is not able to release sufficient insulin. In a later stage, diabetes starts to impact the indirect structure of the body, even the retina. The most common diabetic individuals are infected by retinopathy. In the survey, we could see about 430 million diabetic individuals having the prospect of a visual disability. Diabetic retinopathy (DR) is a delicacy where the retina is hurt by virtue of sap openings in the retina. It happens only when diabetes hurts the infinitesimal deposit inside the retinal core. The sap in the retina structure will leak blood and liquid. The appearance of the integrant on the retina defines the classification, and the periods of diabetic retinopathy are perceived. A trained clinician is required to classify normal or not as it is a long cycle, and the clinician is also needed to check out and examine the dataset diversity of the fundus photographs. One of the fundamental difficulties is early identification, which is vital for treatment achievement. The specific ID of the diabetic retinopathy stage is interesting and requires master human comprehension of fundus pictures. Improvement of the recognition step is pivotal and can help a large number of individuals. Neural networks (NNs) have been successfully used to discover diabetic retinopathy in several contiguous patients.

Here, we proposed one more computation to recognize the retinal veins. The green channel will be chosen for picture investigation to precisely extricate vessels. The discrete wavelet change is utilized to upgrade the picture contrast for viable vessel identification. The directionality component of the multi-structure component strategy makes it a successful device in edge discovery. Hence, morphology administrators utilizing multi-structure components are applied to the upgraded picture to find the retinal picture edges. A short time later, morphological administrators by reproduction dispose of the edges not having a place with the vessel tree while attempting to protect the slight vessels unaltered. To extend the efficiency of the morphological heads by propagation, they were applied using multi-structure components.

Due to their capacity to identify and train the most discriminative features at the pixel level, neural networks, a subset of deep learning, have outperformed traditional machine learning-based techniques for medical imaging segmentation. In this study, we create a method for the automatic segmentation of retinal haemorrhages in the fundus picture using a neural network-based architecture. We use datasets with very high-quality photos tagged pixel by pixel to train neural networks. To teach the network to make judgments by delivering accurate information, the initial step is to search the data.

This paper is organized as follows: Section 2 briefly explains existing works.  Section 3 presents the proposed methodology.  Section 4 discusses feature extraction.  Section 5 describes performance metrics.  Section 6 provides the conclusion.

## 2. Literature Survey

The paper [1] proposed content-based picture recuperation that has been shown to be progressively more supportive for a couple of utilization spaces, from differing media to security. As content-based recuperation was developed, different legitimate applications were revealed to clients for such techniques. Further, lately, plant applications delivered very colossal picture arrangements and a short time later ended up outstandingly mentioning content-based visual resemblance calculation. In this paper, we depict low-level element extraction for visual appearance examination between genetically changed plants for quality articulation studies. The paper [2] explained a database that has various sizes, which may not be handled similarly. Moreover, normalizing the sizes consistently would require further preprocessing before extricating the qualities. The review utilizes the article's meaning of picture and variety correlogram to restore the picture recovery region as an objective region. What is more, to address decayed execution because of variety recovery, the picture shape data is utilized. The characterized region is not altogether affected by foundation tone, so the proposed strategy might have improved and brought about the recovery need. The paper [3] stated that a variety correlogram is a straightforward factual description of a variety of pictures that has been broadly utilized for content-based image retrieval (CBIR) frameworks. To quantify closeness between two pictures utilizing the correlogram, the conventional methodologies utilize the relative distance. In this paper, to further develop the execution of the CBIR frameworks, the inward item metric is utilized to quantify the similitude of pictures rather than the relative distance. Aftereffects of analyses demonstrated that the CBIR utilizing the internal item metric has preferred execution over the one utilizing the relative distance.

The paper [4] presented a substance-based picture recovery framework, called MPEG-7 picture recovery refinement given importance criticism called (MIRROR), created for assessing MPEG-7 visual descriptors and making new recovery calculations. The framework center depends on MPEG-7 trial and error mode (XM) with web-based UI for question-by-picture model recovery. Another consolidated variety range approach for MPEG-7 predominant variety descriptor likeness measure and pertinence criticism is likewise evolved in this framework. A few MPEG-7 visual descriptors are taken on in MIRROR for execution examination purposes. The paper [5] created a content-based image retrieval (CBIR) outline given the edge recognition technique for analysis of diabetic retinopathy. Typical and unusual retinal fundus pictures are exposed to preprocessing techniques to upgrade the edge data. Two distinct strategies, specifically Kirsch layout and Canny edge-based identification methods, are considered for the division of veins. The design and surface-based highlights acquired from portioned pictures are examined. The best highlights for retinal picture recovery are chosen from the quantitative investigation of elements. Similitude matching is done utilizing the Euclidean distance technique, and the recovered pictures are positioned. Recovery productivity is determined by accuracy and review. The outcomes show that the Kirsch format-based edge recognition strategy distinguishes the majority of the veins contrasted with the other technique [6, 7]. A serious level of accuracy and review is noticed utilizing the Kirsch format-based CBIR framework. The Kirsch edge-based location could be valuable in the CBIR framework for the conclusion of retinal irregularities.

## 3. Methodologies

Artificial neural networks are the foundation of the deep learning (DL) class of artificial intelligence (AI) techniques, which are inspired by the structure of the human brain. DL essentially refers to techniques for automatically learning the mathematical representation of the latent and intrinsic relations of the data. Contrary to typical machine learning techniques, deep learning ones learn the proper features directly from the data instead of relying on the development of hand-crafted features, a procedure that may be very time-consuming and labor-intensive. Additionally, when the volume of data grows, DL methods scale significantly better than conventional ML methods. An outline of certain important DL ideas is given in this section.

### 3.1. Existing System

The current framework utilizes classification methods like a retinal grading algorithm (RGA), a fuzzy rule-based characterization framework, and a support vector machine (SVM) algorithm cycle to recognize diabetic retinopathy [8–13]. In this calculation, just the power is being viewed as a serious issue, and a solitary limit is utilized as an incentive for the entire picture. It contrasts the retinal pictures well when there is a justifiable edge of separation between classes. It is exceptionally utilized for the arrangement of the issues in the pictures. In any case, the current calculations have a few disadvantages: the connections between pixels are not being viewed as the calculation is not reasonable for huge informational collections and does not genuinely do well when the informational index has further commotion that the target classes are lapping. It is difficult to track down the ideal angles [14–18]. Along these lines, the inner parts of the retina make the most common way of finding veins troublesome. Edge identification is absurd to anticipate arranging fundus exudates. Responsiveness, particularity, and precision are not anticipated with a superior exhibition of the fundus pictures.

### 3.2. Proposed Methodology: Neural Network Design

The design of the proposed model for detecting diabetic retinopathy consists of four basic tasks, namely, preprocessing, segmentation, feature extraction, and classification. As stated above, the initial fundus image of the retinal eye is preprocessed. Under the preprocessing process, the following steps are performed:

- Color conversion.
- Resizing.
- Filtering.

#### 3.2.1. Color Conversion

In image processing, color conversion is used to convert RGB (red, green, and blue) to grayscale reading. Since RGB has higher complexity, converting it to gray scale increases the intensity, and as a result, efficiency is also increased. The value of the RGB image is 24 bits, while the gray value is 8 bits.

#### 3.2.2. Resizing

Image resizing refers to the scaling of pixels wherein lowering the range of pixels from a picture is facilitated; i.e., it can lessen the time of schooling of a neural community as the larger the range of pixels in a picture, the larger the range of entering nodes that during flip will increase the complexity of the model. It also helps to zoom in on pixels. In case of resizing the picture, it does both reduction and scale-up to satisfy the dimension requirements.

#### 3.2.3. Filtering

The filter we use here is median filter. The median filter approach is utilized for dispensing with the commotion in the contribution of the retinal fundus pictures and signals. The median filter is given in detail within the given input image where the processing area is widely recognized for the preservation of the edges to eliminate the noise.

#### 3.2.4. Decomposition

Wavelets are functions that can be used to subdivide a signal into distinct frequency bands (sub-bands) prior to processing and quantization, as an alternative to transforms like the discrete cosine transform (DCT). The DWT disintegrates an information picture into four parts named LL, HL, LH, and HH. The primary letter means whether a low pass or high pass recurrence activity is utilized to the lines, while the subsequent letter indicates the channel applied to the sections. The estimated part of the first picture makes up the most reduced goal level, LL. Particularly for low piece rate applications, discrete wavelet changes (DWT) based picture coding outperformed regular DCT-based picture coding in terms of insight and sound handling. Accordingly, some notable coders have been proposed to pack pictures or casings handled by DWT effectively. The detailed parts of the other three goal levels offer upward high (LH), even high (HL), and high (HH) frequencies.  Figure 1 shows a 2-level wavelet deterioration of a picture. Dermatologists use medical clinic symptomatic ways to deal with a view of visual differentiation inside the retina as well as changes in the retina's appearance after some time.

In the processing method of input, fundus images use surface examination to catch these visual properties where 2 levels of disintegration and give a multigoal insightful structure for portraying an info picture north of a few recurrence spaces. Because the fundus images are obtained under the scope of conditions, including deferred picture securing arrangements of intensity, and visual focusing, which diversify the blood vessel on the diagnosis, 2 levels of decomposition are profoundly helpful. In the detection of diabetic retinopathy, to get exact data, we utilized the 2D wavelet change. This 2-level decomposition comprises various investigations; however, in our assessment, we use the tree-structured wavelet study to empower low-, center-, and high-recurrence decay by deteriorating both unpleasant and detailed coefficients. The lower recurrence parts of the retinal picture gave data on the impacted region of the fundus picture, which is useful for determination, while the higher repeat crumbling exhaustively offers experiences in regard to the degree of decay and central examination. For this situation, the deterioration of all repeat channels is appealing.

## 4. Feature Extraction

In this survey, GLCM is used to isolate the components. The GLCM limits determine how much time sets of pixels with values got and in a specific spatial connection occur in an image, by producing a GLCM, and after a period removing estimates from this grid to portray an image's surface [19–23]. After the decomposition process, GLCM analysis of the input image is made. The limits determine how habitually a pixel with the richness (dark level) *k* shows up in a particular structural association with a pixel with the worth *l* to fabricate a GLCM. The pixel's value and the pixel's uniformly continuous arrangement define their structural relationship; in any case, it can portray different structural associations. The addition of every component (k, l) is the result of GLCM which shows how many times the pixel with the worth *k* existed in the predetermined structural relationship to a pixel with the worth *l* in the info picture. The size is not entirely settled by the dark levels in the given retinal picture. Obviously, gray co-network scales an image to lessen the number of force values to eight, and yet can change these scales with the Num Levels and Gray Limits settings. The gray co-occurrence matrix can show the deep outline of dim levels in the surface picture. The surface is coarse concerning the picked counterbalance in the event that most of the sections in the GLCM are grouped along the skew.

The gray co-matrix is utilized to work out the initial three qualities in a GLCM, as displayed in Figure 1. The result of GLCM in the figure is portrayed by three types of components:

- Component (1, 5) has the worth 1 because it has a single case of two equally neighboring pixels.
- Component (5, 7) has the worth 2 because there are two occurrences on a level plane nearby pixels.
- Component (2, 1) has the worth 0 because there are no events on a level plane nearby pixels.

Gray co-matrix continues taking care of the data picture, separating the image for other pixel matches (k, l), and keeping the totals while looking at parts of the GLCM.

### 4.1. Parameters of GLCM

Entropy measures picture surface abnormality; when the space co-occasion system for all values is the same, it achieves the base worth [24].

(1) $$\begin{array}{c} S=\sum \;p_{s}\left(x,y\right)\log p_{s}\left(x,y\right)\text{,} \end{array}$$

where *p*_s_ refers to the entropy. Contrast is the primary feature from corner to corner near the portrayal of laziness, which assesses the value of the association and pictures of adjacent changes in the number, reflecting the image clarity and surface of shadow importance [25].

(2) $$\begin{array}{c} \Delta contrast={\left(x-y\right)}^{2}\text{.} \end{array}$$

Correlation coefficient measures the joint probability occasion of the prescribed pixel matches.

(3) $$\begin{array}{c} \rho \left(X,Y\right)=\frac{cov\left(X,Y\right)}{\sigma X}\text{.} \end{array}$$

Homogeneity, commonly known as the inverse difference moment, is a measure of how close components in the GLCM are to the diagonal.

(4) $$\begin{array}{c} H=\sum \sum \left(\frac{p\left(x,y\right)}{\left(1+\left[x-y\right]\right)}\right)\text{.} \end{array}$$

Figure 2 shows the process of feature extraction. Here, in the GLCM feature extraction, firstly, it analyzes retinal fundus input image by convoluting in multilayer by the co-occurrence of the matrix method. Once the convolution is done, the pooling method is examined by conducting another multilayer analysis. After pooling, the classification algorithm is used to detect diabetic retinopathy by the fully connected method.

### 4.2. NN Process and Detection

A hub is only where registering occurs about displayed after a neuron in the human brain that fires when sufficiently animated. A hub joins information input with a bunch of coefficients or loads that either enhance or hose that information, relegating significance to inputs about the objective the calculation is attempting to learn the right characterizing input information is made a sum of such information weight items is then sent through a hubs purported enactment work which decides if and how far the sign ought to go through the organization to influence the end result. A hub layer is a bunch of neuron-like fasteners and turns 0/1 as information goes through the organization beginning with the main study layer. It acknowledges your message. The feedback from the following layers is also included in each layer's output. We attach importance to entering highlights by consolidating the model's configurable loads with input key attributes of how the brain network classifies and gathers information. A model is an assortment of loads that endeavors to address information's relationship to ground truth identifiers to completely comprehend the information's design either by the being or finishing the state. Models normally begin horrendously and improve when the brain organization's boundaries are refreshed [12, 13].

This is on the grounds that a brain network is made with no information. It has no clue about which loads and inclinations will successfully make an interpretation of the data into exact estimates. It should start with an estimate and afterward steadily work on its theories as it improves its slipups. A brain network is considered to be a more modest form of the logical technique, which includes testing hypotheses and attempting once more, albeit with a blindfold on. Or, on the other hand, similar to a baby, it begins knowing very little and steadily figures out how to tackle hardships on the planet through openness to life experience. Data is the main information that brain networks have. Here is a quick explanation of what happens when you learn with the most basic design, a feed-forward neural network. The network receives input. The parameters, or weights, translate the input into a set of final guesses made by the network [14–22].

(5) $$\begin{array}{c} Weight*Input=Guess\text{.} \end{array}$$

When you use weighted input, you get a prediction about the input. The neural network then compares its assumption to the data's ground truth (D_GT_).

(6) $$\begin{array}{c} D_{GT}-E=NN_{Guess},where\;E\;is\;an\;error\text{.} \end{array}$$

The mistake is the distinction between the organization's estimate and the ground truth division. It ascertains the mistake and checks it back through its type, changing loads to the degree that they prompts it.

(7) $$\begin{array}{c} Adjustment=NN_{Error}*Load\;percentage\;to\;error\text{.} \end{array}$$

The above numerical articulations represent the major activities that show how the brain organizes is as follows: assessing feed, figuring misfortune, and refreshing the mode which rehash the above venture process. A cerebrum network is a self-redressing input circle that prizes stacks that help it with making the right gauges and rebukes stacks that cause it to commit mistakes.

## 5. Performance Measurement

Numerous presentation estimations are applied to deep learning strategies to quantify their grouping execution. Precision, responsiveness, particularity, and area under the ROC curve are standard deep learning measurements. The level of strange pictures named unusual is called responsiveness, while the level of typical pictures classified as expected is called explicitness. The level of accurately classified photographs is known as precision. Coming up next are the conditions of estimation.

(8) $$\begin{array}{c} {Specificity}_{p}=\frac{{TA}_{b}}{\left({TA}_{b}\right)+FN}\text{,}\\ {Sensitivity}_{P}=\frac{TN}{\left(TN+{FA}_{b}\right)}\text{,}\\ {Accuracy}_{p}=\frac{{TA}_{b}+TN}{\left({TA}_{b}+TN+{FA}_{b}+{FA}_{b}\right.}\text{,} \end{array}$$

where *p* is the performance. True normal (TN) is one of the quantities of poor pictures that are delegated an infection genuine. True abnormal (TA_b_) is the quantity of ordinary pictures that are delegated typical while false normal (FN) is the quantity of typical pictures that are named an infection false. Abnormal (FA_b_) is the level of execution estimates used in the tests related to the ongoing work are based on how many bad photographs are named as being usual.

Figure 3 shows the comparison of defined parameters.  Figure 4 shows the output of performance measurements.

Due to their superior power and capacity to automatically extract features as compared to machine learning-based approaches, deep learning-based systems have grown in popularity, as shown by prior works. Deep learning additionally enables precise localization of the retinal borders. The only drawback is that it requires lengthy and challenging training.

Existing diabetic retinopathy methods contain variables like sensitivity, specificity, and accuracy that are substantially lower than the output of the necessary elements for this project. Sensitivity is 80.21%; specificity and accuracy are not stated for the moat operator approach. The sensitivity, specificity, and accuracy of the support vector machine are higher than those of the moat operator technique, which are, respectively, 82.5%, 88.9%, and 82%.

In contrast to the aforementioned techniques, fuzzy rule-based classification has accuracy of 92.4%, specificity of 94.29%, and sensitivity of 92.44%. However, the non-detection of entropy, energy, contrast, homogeneity, and correlation coefficient in retinal pictures presents a significant issue. The objective is to raise accuracy, specificity, and sensibility. The proposed model has the following performance metrics for detecting diabetic retinopathy: 96.1538% sensitivity, 95.6522% specificity, and 95.9184% accuracy. Therefore, the main objective of the task is to locate the afflicted portions of the retina in the early stages to prevent the affected people from going blind as well as to help doctors in a more accurate, regular, and quick manner using the identification and percentage-based methodologies.

## 6. Conclusions

The result of the project is obtained when the image processing techniques are executed on the input fundus image. The output experiments that are performed in this project are done in MATLAB. MATLAB 2021 version is required for this project. The vital revelations of the picture pre-handling, time intricacy, and classing results are discussed. Furthermore, differentiation of the paperwork is put forward against regular strategies. Our project depends on a GUI stage. At first, the graphical UI shows the input picture of the patient from its point of interaction. The preprocessing is performed by changing the RGB picture into a gray image and resizing the changed picture; afterward, a filtering medium is utilized to eliminate undesirable disturbance from the picture and give the result in the form of a histogram picture. The decomposition of the fundus image is made by the discrete wavelet transform. Once the decomposition is finished, feature extraction of the fundus image is examined by the gray level co-occurrence matrix (GLCM) for all the pictures in the training dataset by the neural network algorithm, and later these metrics will be utilized to independently compare the results with those in the information picture. The outcome shown that the future steps to be completed for the individual by providing the performance metrics include sensitivity, specificity, and accuracy regardless of whether the person is affected by diabetic retinopathy or not. This research paper mainly focuses on detecting diabetic retinopathy present in the blood vessels of the retina using neural network of deep learning. The input fundus image and DR database are used to test the NN classifier. Here, they will test and determine whether the diabetic retinopathy classification is normal or abnormal. There are existing methods of diabetic retinopathy which have much less sensitivity, specificity, accuracy, etc. compared to the output of the required factors in this project. In the moat operator method, the sensitivity is 80.21%, specificity is about 70%, and accuracy is not reported. In the support vector machine, the sensitivity, specificity, and accuracy are increased compared to those of the moat operator method which are about 82.5%, 88.9%, and 82%.

When compared to the above methods, fuzzy rule-based classification has sensitivity of 92.44%, specificity of 94.29%, and accuracy of 92.4%. But there is a big challenge here, that is, the non-detection of entropy, energy, contrast, homogeneity, and correlation coefficient in retinal images. However, the aim is to improve sensibility, specificity, and accuracy. The proposed model detects diabetic retinopathy with a sensitivity of 96.1538%, specificity of 95.6522%, and accuracy of 95.9184%. Subsequently, the primary goal of the task is to identify the affected areas of the retina in the early stages to prevent the blindness of the affected individuals and also to assist doctors in a more reliable, consistent, and faster manner by the identification and percentage-based techniques.

## Figures and Tables

**Figure 1:** Representation of proposed methodology.

**Figure 2:** Process of feature extraction.

**Figure 3:** Comparison of defined parameters.

**Figure 4:** Output of performance measurements.

## Data Availability

The datasets used and/or analyzed during the current study can be obtained from the corresponding author on reasonable request.

## References

[1] Sinthanayothin C., Boyce J. F., Williamson T. H. (2002). Automated detection of diabetic retinopathy on digital fundus images. *Diabetic Medicine*.

[2] Acharya U. R., Lim C. M., Ng E. Y. K., Chee C., Tamura T. (2009). Computerbased detection of diabetes retinopathy stages using digital fundus images. *Proceedings of the Institution of Mechanical Engineers - Part H: Journal of Engineering in Medicine*.

[3] Afrin R. (2019). *Automatic detection and classification of diabetic lesions for grading diabetic retinopathy using fuzzy rule-based classification system*.

[4] Martinez M. E. P., Hughes A. D., Thom S. A., Parker K. H. Improvement of a retinal blood vessel segmentation method using the insight segmentation and registration toolkit (ITK).

[5] Mendonc A. M., Campilho A. (1213, Sep). Segmentation of retinal blood vessels by combining the detection of centerlines and morphological reconstruction. *IEEE Transactions on Medical Imaging*.

[6] Yalin N., Alver S., Uluhatun N. Classification of retinal images with deep learning for early detection of diabetic retinopathy disease.

[7] Kshirsagar P. R., Chippalkatti P. P., Karve S. M. (2018). Performance optimization of neural network using GA incorporated PSO. *Journal of Advanced Research in Dynamical and Control Systems*.

[8] Kumar Kilari E., Putta S. (2016). Delayed progression of diabetic cataractogenesis and retinopathy in STZ-induced diabetic rats. *Cutaneous and Ocular Toxicology*.

[9] Kauppi T., Kälviäinen H. Simple and robust optic disc localization using colour decorrelated templates.

[10] Mirajkar S., Pati M. M. (2013). Feature extraction of diabetic retinopathy images. *International Journal of Computer Application*.

[11] Dua S., Kandiraju N., Thompson H. W. Design and implementation of a unique blood-vessel detection algorithm towards early diagnosis of diabetic retinopathy.

[12] Sathawane N. K. S., Kshirsagar P. (2014). Prediction and analysis of ECG signal behaviour using soft computing. *International Journal of Renewable Energy Technology*.

[13] Kshirsagar P. (2021). Operational collection strategy for monitoring smart waste management system using shortest path algorithm. *Journal of Environmental Protection and Ecology*.

[14] Rathish C. R., Rajaram A. (2016). Efficient path reassessment based on node probability in wireless sensor network. *International Journal of Control Theory and Applications*.

[15] Rahamat S. B., Sharma C., Sayeed F. (2022). Implementation of reliability antecedent forwarding technique using straddling path recovery in manet. *wireless communications & mobile computing (online)*.

[16] Indira D. N. V. S. L. S., Ganiya R. K., Ashok Babu P. (2022). Improved artificial neural network with state order dataset estimation for brain cancer cell diagnosis. *BioMed Research International*.

[17] Ganesh P., Naidu G. B. S. R., Swaroopa K. (2022). Implementation of hidden node detection scheme for self-organization of data packet. *Wireless Communications and Mobile Computing*.

[18] Dinesh M., Arvind C., Sreeja S. M. (2022). An energy efficient architecture for furnace monitor and control in foundry based on industry 4.0 using IoT. *Scientific Programming*.

[19] Mahalakshmi K., Kousalya K., Shekhar H. (2021). Public auditing scheme for integrity verification in distributed cloud storage system. *Scientific Programming*.

[20] Divakaran J., Malipatil S., Zaid T. (2022). Technical study on 5G using soft computing methods. *Scientific Programming*.

[21] Gobinathan B., Mukunthan M. A., Surendran S. (2021). A novel method to solve real time security issues in software industry using advanced cryptographic techniques. *Scientific Programming*.

[22] Shitharth S., Meshram P., Kshirsagar P. R., Manoharan H., Tirth V., Sundramurthy V. P. (2021). Impact of big data analysis on nanosensors for applied sciences using neural networks. *Journal of Nanomaterials*.

[23] Kshirsagar P. R., Manoharan H., Shitharth S., Alshareef A. M., Albishry N., Balachandran P. K. (2022). Deep learning approaches for prognosis of automated skin disease. *Life*.

[24] Chandan R. R., Kshirsagar P. R., Manoharan H. (2022). CCC publications substantial phase exploration for intuiting covid using form expedient with variance sensor. *International Journal of Computers, Communications & Control (IJCCC)*.

[25] Kshirsagar P. R., Manoharan H., Kasim S. (2022). Expedite quantification of landslides using wireless sensors and artificial intelligence for data controlling practices. *Computational Intelligence and Neuroscience*.

